# Coronary Vessel Segmentation by Coarse-to-Fine Strategy Using U-nets

**DOI:** 10.1155/2021/5548517

**Published:** 2021-04-09

**Authors:** Le Nhi Lam Thuy, Tan Dat Trinh, Le Hoang Anh, Jin Young Kim, Huynh Trung Hieu, Pham The Bao

**Affiliations:** ^1^Information Science Faculty, Sai Gon University, Vietnam; ^2^Industrial University of Ho Chi Minh City, Vietnam; ^3^Electronics and Computer Engineering Department, Chonnam National University, Republic of Korea

## Abstract

Each level of the coronary artery has different sizes and properties. The primary coronary arteries usually have high contrast to the background, while the secondary coronary arteries have low contrast to the background and thin structures. Furthermore, several small vessels are disconnected or broken up vascular segments. It is a challenging task to use a single model to segment all coronary artery sizes. To overcome this problem, we propose a novel segmenting method for coronary artery extraction from angiograms based on the primary and secondary coronary artery. Our method is a coarse-to-fine strategic approach for extracting coronary arteries in many different sizes. We construct the first U-net model to segment the main coronary artery extraction and build a new algorithm to determine the junctions of the main coronary artery with the secondary coronary artery. Using these junctions, we determine regions of the secondary coronary arteries (rectangular regions) for a secondary coronary artery-extracted segment with the second U-net model. The experiment result is 76.40% in terms of Dice coefficient on coronary X-ray datasets. The proposed approach presents its potential in coronary vessel segmentation.

## 1. Introduction

In all living mammal species, including humans, blood vessels inside the body are highly organized and complex, ensuring that blood flows unidirectionally on vessel branches. Localization, segmentation, and visualization of blood vessels from X-ray angiograms are highly necessary and useful in various medical diagnoses. Based on the blood vessel width, reflectivity, and abnormal branching, we can determine symptoms of vessel diseases such as stenosis, vascular malformation, and atherosclerosis. By using the X-ray angiogram, medical experts or doctors manually detect and delineate the blood vessels. However, this process is time-consuming and challenging in the cases of enormous number of X-ray angiograms and small and thin vessel structures. Hence, it is highly necessary to develop automatic and accurate blood vessel detection and segmentation methods from angiograms. Many related works conducted the coronary vessel segmentation based on the weak contrast between the coronary arteries and the background, strong overlapping shadows of the bones, nonuniform illumination in X-ray angiogram, small and thin vessel branches, complex shape of the vessel tree, and/or other body tissues [1, 2]. These factors can decrease the accuracy of segmentation results.

The improvements in coronary vessel enhancement and segmentation algorithms can be divided into six main categories, such as pattern recognition approaches, model-based approaches, tracking-based approaches, artificial intelligence-based approaches, neural network-based approaches, and miscellaneous tube-like object detection approaches [2]. Liao et al. [3] applied an enhanced multiscale approach to extract 2D coronary artery central lines from X-ray projection images. Authors introduced the 3D symbolic reconstruction based on an energy minimization problem incorporating a soft epipolar line constraint and a smoothness term. The nonlinear anisotropic filtering [4] approach performs anisotropic smoothing without blurring the vessel edges on the local orientation. Hessian-based multiscale filtering [5–8] has been proposed for vessel enhancement. In this technique, an input image is filtered by the derivatives of a Gaussian at multiple scales. Then, the Hessian matrix is analyzed at each pixel in the filtered image to determine the structures' local shape. However, due to the second-order derivatives, the Hessian-based approaches are highly sensitive to noise. Furthermore, this approach led to suppressing junctions, as junctions are characterized similarly to the blob-like structures.

In [6], the authors proposed a filter model based on the regularized gradient vector correlation matrix to avoid the need for second-order derivatives. However, this technique faces the same limitations as Hessian-based filters in finding small and low-contrast vessels when dealing with angiography images, which are noisier and suffer from nonuniform illumination. Truc et al. [7] introduced a new framework for vessel enhancement by applying the directional information present in an image. The input images are first decomposed by a decimation-free directional filter bank (DDFB) into a set of directional images. Distinct appropriate enhancement filters are then used to enhance vessels in the respective directional images. Finally, the enhanced directional images are recombined to generate the output image with enhanced vessels. Although this approach is still noise-sensitive, it reveals the small vessel network and avoids junction suppression. Trinh et al. [8] introduced a hierarchical approach to extract coronary vessels from an X-ray angiogram. They applied the DDFB and Homographic Filtering (HF) since they are suitable for strengthening the vessels at different orientations and radii. To obtain the main and small coronary vessels in various sizes, they used a coarse-to-fine strategy for iterative segmentation based on the Otsu algorithm.

Recently, deep learning approaches have been applied for medical image segmentation and analysis [9–13]. These new powerful techniques based on convolutional neural networks (CNNs) lead to high performance in the field of medical imaging for segmentation without expert knowledge. Many studies confirm that deep learning models outperform traditional medical segmentation systems. In [10], authors developed a successful and well-known network based on the CNN, named as U-net, for biomedical image segmentation. The network architecture consists of two paths: encoder and decoder. The encoder is a contraction stack of convolutional layers used to capture the context of input images. After each convolutional layer, a rectified linear unit (ReLU), max pooling, and dropout layers are added. The decoder is an expansive path that is used to enable precise localization by using transposed convolutions. In the decoder, the final layer is used to map the feature vector to the binary prediction (i.e., vessel vs. nonvessel). The U-net requires the inputs as 2D image patches and returns the 2D segmentation probability map for each given patch. Milletari et al. [11] introduced a V-net architecture that adopts a volumetric CNN for prostate segmentation from MRI. Similar to U-net, V-net induced two paths. The first path (left path) of the V-net consists of a compression path. The second one (right path) decompresses the input image until its original size is reached. Holistic-net [12] was proposed for brain tumor segmentation. It is a combination of holistic CNNs and generalized Wasserstein Dice scores for multiclass segmentation. In [13], a graph neural network (GNN) is proposed to learn global vascular structures in medical images. The authors combined the GNN into a unified CNN architecture to learn not only local appearances but also the global structures of vessels.

Deep learning-based automated ventricle segmentation methods are summarized in the research [14]. Authors [15] developed a novel encoder-decoder deep network algorithm to exploit 2D + *t* sequential images' contextual information in a sliding window. The encoder extracts the temporal-spatial features. The skip connection layers subsequently fuse these features and deliver them to the corresponding decoder stages. The decoder employed the channel attention mechanism. In [16], the authors proposed a nested encoder-decoder architecture named T-Net. T-Net consists of several small encoder-decoders for each block constituting a convolutional network. They evaluated T-Net by segmenting only three main vessels in coronary angiography images and archive the Dice similarity coefficient score of 88.97%. In the research [17], the blood vessels are segmented from both the coronary angiogram and the retinal fundus images using a single VSSC Net after performing the image-specific preprocessing. The VSSC Net consists of two-vessel extraction layers with additional supervision on top of the base VGG-16 network. The VSSC Net attains average AUC values of 0.98205 across the target datasets. Authors [18] proposed a novel weakly supervised training framework to alleviate the annotator's burden by learning from noisy pseudo labels generated from automatic vessel enhancement instead of fully manual annotation. Their annotation-refining self-paced learning framework (AR-SPL) corrects the possible errors using suggestive annotation. Experiments confirm that their proposed framework largely reduced annotation cost and Dice score of 82.09%. Another study proposed an automated prostate MRI data segmentation using bicubic interpolation with improved 3D V-Net. Two clinical prostate-MRI data datasets were used to evaluate the model's effectiveness with the manual delineations available as the ground truth [19]. The segmentation result is 98.29% of average accuracy and 0.9765 of Dice metric.

With the supportive goal of interpreting pathophysiological processes and clinical decision-making, the study [20] developed a multiview recurrent aggregation network (MV-RAN) for the echocardiographic sequence's segmentation with the full cardiac cycle analysis. Experiments were conducted on spatial-temporal (2D + *t*) datasets of multicenter and multiscanner clinical studies. Compared to other studies, the research [20] achieved results of 0.92 Dice score.

This study proposes a novel hierarchical approach to extract coronary vessels from X-ray coronary angiographic images. We use a coarse-to-fine strategy for iterative segmentation based on the U-net model to segment the coronary vessels in various sizes as follows:

- We use U-net to segment the main and large blood vessels
- We propose a new approach to extract junctions from vascular trees and detect small vessel regions based on the main information from extracted vessels
- We apply the region-based U-net segmentation to locate and obtain the small vessels

## 2. Materials and Methods

In this section, we describe the proposed hierarchical approach in detail. As illustrated in Figure 1, our proposed framework includes tree main steps: preprocessing, extracting the large coronary vessels, and extracting the small ones.

The preprocessing procedure is applied to remove high-frequency noise and also enhance the contrast of X-ray coronary angiographic images. We first apply a Gaussian filter to smooth the vessel image. The Gaussian filter is low-pass filtering that is used to reduce high-frequency noise in order to make our vessel segmentation more accurate. In our study, we use Gaussian smoothing to detect false edges or artifacts (not small artery fragments) due to noises and reduce their effect on the input. In addition, a histogram equalization method [21] is applied to adjust the contrast of images.  Figure 2 shows our preprocessing process.

In the next step, we apply a coarse-to-fine strategy for iterative segmentation. Particularly, we segment regions that include the main coronary vessels based on the high-contrast pixels. The main coronary vessels include features such as vascular tree and junctions. Subsequently, we use coarse information extracted in the previous step to detect the small vessels that often have low contrast and are affected by noises. We describe each step of the proposed technique in detail in the following sections.

### 2.1. Large Vessel Extraction Based on U-net

In this section, we describe a method to extract vessels by using U-net and the coarse-to-fine segmentation strategy.  Figure 3 shows a block diagram of the vessel's extraction.

The U-net model is proposed for biomedical image segmentation [10]; as shown in Figure 4, the network architecture consists of encoder and decoder paths. The encoder is a contraction path that captures the context in the input image. The decoder is an expansive path that applies transposed convolutions to enable precise localization. In the decoder, the final layer maps the feature vector to the binary outputs such as vessel or nonvessel. The U-net receives the inputs as 2D image patches and returns the 2D segmentation probability map for each given patch.

The U-net uses the loss function as the cross-entropy function shown as follows:

(1) $$\begin{array}{c} J=-\underset{x\in \Omega }{\sum }w\left(x\right)\log\left(p_{l\left(x\right)}\left(x\right)\right), \end{array}$$

where *p*_*l*(*x*)_ is the soft-max function defined by *p*_*l*(*x*)_ = exp(*a*_*l*_(*x*))/(∑_*l*′=1_^*L*^exp(*a*_*l*′_(*x*))) , where *a*_*l*_(*x*) is an activation in feature channel *l* at the pixel position *x* ∈ *Ω* with *Ω* ⊂ *Z*^2^, *l* : *Ω* → {1, ⋯, *L*} is the true label of each pixel *x*, and *L* denotes the number of classes.

The weight map is computed as

(2) $$\begin{array}{c} w\left(x\right)=w_{c}\left(x\right)+w_{0}\cdot \exp\left(-\frac{{\left(\left(d_{1}\left(x\right)+d_{2}\left(x\right)\right)\right)}^{2}}{2\sigma^{2}}\right), \end{array}$$

where *w*_*c*_ : *Ω* → *R* denotes the weight map to balance the class frequencies, *d*_1_ : *Ω* → *R* is the distance to the border of the nearest cell, and *d*_2_ : *Ω* → *R* denotes the distance to the border of the second nearest cell. In experiments, we set *w*_0_ = 10 and *σ* = 5 pixels following the related research [10].

In this study, the original input images and their corresponding segmentation labeling (or ground truth segmentation) are used to train U-net for extracting the large vessels. For a test case, the input image is required for the U-net model and returns a 2D segmentation probability map.  Figure 5 presents an example of U-net segmentation for large vessels. We can realize that the U-net model can obtain a good performance for large vessel segmentation because of its high contrast to the background. However, the model performance is limited for small vessels.  Figure 5 illustrates that some small vessels are disconnected or broken up vascular segments due to their low contrast to the background and thin structures. Subsequently, to overcome this problem, we propose a coarse-to-fine algorithm-based U-net for detecting and extracting small and thin blood vessels.

### 2.2. Small Vessel Extraction Based on Coarse-to-Fine Algorithm-Based U-net

In the previous section, we represent the U-net approach to extract the main coronary vessels. However, it cannot reveal well the small vessels due to their blurring and low contrast compared with the background. To solve this problem, as shown in Figure 6, we use the information of the main extracted vessels and propose a new method to extract junctions on the vascular tree and extract small regions that included small vessel branches. Then, we apply a region-based U-net approach to segment small vessels based on a coarse-to-fine mechanism.

The branching geometry and junctions of the blood vessel tree are challenges in applying the coarse-to-fine U-net framework for vessel segmentation. The Zhang-Suen thinning algorithm [21] can be applied to extract the skeleton or central line of the main vessels. However, after segmentation, thin broken blood vessels may appear due to low contrast or low signal-to-noise ratio, leading to reduced performance. Therefore, we introduce an improved Zhang-Suen thinning algorithm to connect small broken blood vessels. We summarize this approach in Algorithm 1, and Figure 7 displays the result after applying this algorithm.  Figure 8 presents the blood vessel's central line result based on an improved Zhang-Suen thinning algorithm.

The start, end, and junction nodes of the blood vessels are determined based on the central line of the large vessel segmentation result. In an X-ray angiogram, because of the huge number of vessel branches, it is necessary to distinguish each blood vessel branch.  Algorithm 2 describes a method to detect important nodes in the blood vessel. Given a central line image (skeleton binary image) of the large vessel segmentation result (output from Algorithm 1), object pixels (foreground) will have the value 1 (belonging to the blood vessel tree) and background pixels will have 0. For each pixel in the binary image, we classify each pixel (*i*, *j*) belonging to a particular label. Specifically, background pixels that have the value of 0 is classified into class 0 (or label 0). These background pixels are ignored while finding the important nodes. Consider object pixels as the foreground, whether an object pixel has exactly two neighbour object pixels, this object pixel is considered a midpoint in the skeleton image (not the start, end, or junction points) and it is classified into class 1 and is ignored while finding the important nodes. Finally, an object pixel that has exactly one neighbour object pixel is considered start and end nodes and is classified into class 2; the object pixel has more than two neighbour object pixels, and it is a junction node and is classified into class 2. For each object pixel (*i*, *j*) in the skeleton image and having label 2, we find all neighbour object pixels of pixel (*i*, *j*) that were classified into class 2 and then calculate their centroid point. The centroid points are considered the important nodes.  Figure 9 demonstrates the determined nodes in the blood vessel tree.

Usually, the small vessels from an X-ray angiogram are blurring low-contrast images. It is difficult to extract large and small vessels simultaneously. For that reason, a local region-based segmentation approach should be used to extract the small ones. Based on the idea from local thresholding, we apply a region-based U-net to segment these small vessels. This approach helps reduce the effect of changing in grayscale values between the vessels and the background compared to the global approach. For each node in the blood vessel tree, we will construct a window between nodes *i* and *j*. The width (*w*) and height (*h*) of the window are described by

(3) $$\begin{array}{c} w=\left|\left(x_{i}-x_{j}\right)\right|+\text{bias}, \end{array}$$

(4) $$\begin{array}{c} h=\left|\left(y_{i}-y_{j}\right)\right|+\text{bias}. \end{array}$$

In our experiment, we select a bias of 20 pixels for obtaining small vessels near node *i*. The proposed approach focuses on determining regions of small blood vessels as summarized in Algorithm 3.  Figure 10 describes an example of a local region that includes small vessels. In the local region, there exists a large vessel with high intensity and high contrast to the background compared to small vessels. Thus, we remove the effect of the large vessel in the window and then apply contrast adjustment based on image processing to areas that include the small vessels.  Figure 11 presents a contrast enhancement based on image processing in the small region. Additionally, we apply the region-based U-net approach to segment these small vessels.

## 3. Results and Discussion

### 3.1. Dataset

All of the experiments were conducted on the X-ray angiogram database of the coronary vessel, which was collected and supported by local hospitals. The database contains 48 different vessel images corresponding to two categories: D1 and D2. The size of each image is 512 × 512 pixels, with 256 gray levels per pixel. The D1 dataset consists of 20 images that obtain a direct front view of the coronary vessels. The D2 dataset includes 28 images taken from four different angles of the coronary vessels [8].

Our dataset is divided into 40 images for training and 8 images for testing. During the training process, we use data augmentation methods to enhance the performance of the segmentation result. This method allows the network to become invariant and robust to certain transformations when the size of the training set is limited. For example, rotation, flip, and shear operators are usually used for convolutional neural networks and yield the desired invariance and robustness properties of the resulting network. In our experiment, the augmentation was applied using the ImageDataGenerator function implemented in Keras.

### 3.2. Experimental Environment

In the experiments, we use the software MIPAR of Sosa [22] to create ground truth in order to evaluate the performance of the segmentation algorithm. We compute the Dice similarity coefficient [23] between binary segmentation results and the ground truths to evaluate the accuracy of our system.  Figure 12 shows a sample image and its ground truth. Our experiments are implemented on an Intel® Xeon® E5-2630, CPU @ 2.3GHz with 128 GB RAM, 4 GPU NVIDIA Geforce GTX 1080Ti - Vram 11 GB (CUDA 6.1). The average runtime of the proposed algorithm to be applied to each image is 66.67 ms. In the large blood vessel extraction procedure, we use the U-net model with 64 filters for the first convolutional layer, followed by the ReLU activation function, we set the learning rate of 1*e* − 4, and the sigmoid function is used as the final activation function. The training process of region-based U-net is similar to that of the original U-net model. The region-based U-net is a small version of the original U-net. Particularly, it is modified with a small number of filters of 16 for the first convolutional layer to deal with small input images (including small vessel regions). The small vessel regions from the same original training set are used to train a region-based U-net model.

In the small blood vessel extraction procedure, we use the U-net model with 16 filters for the first convolutional layer, followed by the ReLU activation function, we set the learning rate of 1*e* − 4, and the sigmoid function is applied for the final activation function.

## 4. Results

This research investigates the coronary vessel segmentation performance based on the coarse-to-fine strategy-based U-net for iterative segmentation comprising other approaches.  Figure 13 illustrates a segmentation result of the proposed approach. We found through experimental analysis that our method segments the large coronary vessels significantly. The performance of size-independent coronary vessel segmentation attains 80.17%. Besides, our method reveals a large number of small and thin blood vessels. Finally, the proposed approach obtains the average of the performance of coronary vessel segmentation of 76.40%. We also compare the proposed approach's performance with the baseline U-net and the other techniques in [7, 8] on our database.  Figure 14 shows a comparison of segmentation results.  Table 1 describes a summary of the coronary vessel segmentation performance in terms of the Dice coefficient. The experimental results are described as mean ± standard deviation.

From Figure 14 and Table 1, we realize that our method using the hierarchical approach based on deep learning and coarse-to-fine strategy obtains better segmentation results and outperforms the standard approaches. In Figure 14, we can realize that the DFB-based segmentation [7] leads to more artifacts and fails to enhance small vessels compared to our approach correctly. Furthermore, it cannot detect the small vessels that have low intensity and large vessels with missing parts. Our method detects the large and small vessels at the same time; even in the case of existing large difference in intensity between the large vessels (which are high-contrast objects) and the small vessels (which are low-contrast objects), the DFB-based method cannot significantly extract small vessels. The proposed method in [8] can extract large blood vessels very well, but it leads to missed extraction of small and thin vessels and vessels with low contrast to the background. Experimental analysis indicated that the baseline U-net yields higher accuracy than the traditional DFB and Otsu approach. The U-net can obtain very high accuracy for the main vessels. However, it also leads to missed extraction of small ones. Our proposed method-based U-net and coarse-to-fine strategy-based segmentation provide the optimal performance.

Our method is proposed to overcome the problem by separately detecting the large vessels and small vessels based on a hierarchical technique via the U-net model. Because we consider that the large vessels always have high contrast to the background than the small vessels, the U-net model is suitable for extracting them. The coarse-to-fine strategy-based segmentation guarantees that the method can correctly extract the large vessels. In the small vessel extraction stage, we first reduce the effect of large vessels and make a contrast enhancement on the region that includes small vessels. This deals with the low-contrast problem on small vessel regions. When the small vessel regions have increased the contrast, they were easily detected and segmented by U-net. This is significant to extract small vessels. The experimental results show that our method overcomes the limitations of the standard approaches, such as small vessel intensity and noise sensitivity. It also performs better on real angiography images.

However, most errors occurred while processing small vessels. These errors cause contrast enhancement based on an image processing technique and quality of small images. In particular, the traditional contrast enhancement approach has errors due to the background enhancement with fewer artifacts. In our cases, several small vessel images are affected by illumination and noises, such as low-light conditions and low contrast. The traditional contrast enhancement approach cannot deal with all problems leading to reducing the accuracy of our segmentation system.  Figure 15 shows a small vessel image affected by illumination and contrast enhancement. Some small vessel branches are missing.

Our research contains other limitations rather than the dependence on traditional methods for contrast enhancement. There is a limitation in the number of public datasets of X-ray angiograms of the coronary vessels. Researchers have limited access to X-ray angiograms of coronary vessel data. In addition, this research is a proof-of-concept study and limited by the size of the dataset. Our dataset is considered small for developing a completed medical image-based deep learning application. Medical image segmentation-based deep learning requires sufficient data to obtain higher accuracy than traditional systems.

## 5. Conclusions

We introduce an improved coronary vessel segmentation technique by a hierarchical approach based on the coarse-to-fine strategy for iterative segmentation using U-net architecture. Our method not only segments the main blood vessels but also locates and extracts the small and thin vessel branches. Through experiments results, it has been confirmed that our proposed method is effective and can enhance the performance of vessel segmentation. However, small vessel images are missing due to enhancing the background with fewer artifacts when these images are applied to contrast enhancement based on the traditional image processing technique. In the future, we intend to improve the results for small and thin vessels by exploiting the superpixel-based deep learning approach to enhance the quality of small vessel image and explore other deep learning frameworks for coronary vessel segmentation and an extended method to deal with 3D images.

## Figures and Tables

**Figure 1:** An illustration of the proposed method.

**Figure 2:** Preprocessing process.

**Figure 3:** Vessel's extraction based coarse-to-fine segmentation.

**Figure 4:** Illustration of the U-net architecture [10].

**Figure 5:** An example of U-net segmentation result.

**Figure 6:** A block diagram for small vessel extraction.

**Figure 7:** An example of connecting the nearest the central lines: (a) input image and (b) image after connecting the nearest central lines (reproduced from Trinh et al. 2019 [under the Creative Commons Attribution License/public domain]).

**Figure 8:** Results of the central lines of blood vessels based on the improved Zhang-Suen thinning algorithm. Input image. Result of the baseline Zhang-Suen thinning algorithm. Result of the improved Zhang-Suen thinning algorithm.

**Figure 9:** An example of nodes (starting, end, and junction points) in the blood vessel tree.

**Figure 10:** An example of a region constructed between two nodes.

**Figure 11:** An example of contrast enhancement in the region analysis: (a) input image and (b) result from contrast enhancement (reproduced from Trinh et al. 2019 [under the Creative Commons Attribution License/public domain]).

**Figure 12:** Ground truth of an X-ray angiogram image.

**Figure 13:** Segmentation result of the proposed approach: (a) input image; (b) ground truth; (c) segmented blood vessels.

**Figure 14:** Comparison of the segmentation results: (a) input image; (b) result in [7]; (c) result in [8]; (d) result of our method.

**Figure 15:** Under segmentation error of small vessel image due to the effect of illumination: (a) input image; (b) contrast enhancement image; (c) result using U-net; (d) result of our method.

**Algorithm 1:** Vessel central line extraction from a binary image.

**Algorithm 2:** Detecting important nodes in the blood vessel tree.

**Algorithm 3:** Small blood vessel region detection.

**Table 1:** Performance comparison of the coronary vessel segmentation in terms of Dice coefficient.

Method	Dice coefficient (%)
DFB-based segmentation [7]	45.50 ± 1.31%
Coarse-to-fine-based DFB and Otsu [8]	71.34 ± 0.80%
Baseline U-net [10]	73.64 ± 1.32%
Proposed approach	76.40 ± 1.02%

## Data Availability

We use private data from the hospital.
